The article "Acute Effects of Different Intensities of Cycling Acute Exercise on Carotid Arterial Apparent Elasticity and Hemodynamic Variables" was published in 2020. Journal: Biomed Res Int.

# Acute Effects of Different Intensities of Cycling Acute Exercise on Carotid Arterial Apparent Elasticity and Hemodynamic Variables

**DOI:** 10.1155/2020/9027560

**Published:** 2020-11-08

**Authors:** Bing-Yi Shen, Hai-Bin Liu, Ling Cao, Kai-Rong Qin

**Affiliations:** ^1^School of Kinesiology and Health Promotion, Dalian University of Technology, Dalian 116024, China; ^2^School of Optoelectronic Engineering and Instrumentation Science, Dalian University of Technology, Dalian 116024, China

## Abstract

**Background:**

Cardiovascular disease (CVD) is closely related to arterial elasticity and hemodynamics. Exercises have been reported to immediately decrease arterial apparent elasticity and regulate hemodynamic variables. However, the relationship between them and exercise intensity remains elusive. The purpose of this study was to determine the acute effects of different intensities of acute cycling exercise on carotid arterial apparent elasticity and hemodynamics.

**Methods:**

32 healthy men (age: 19.4 ± 0.6 years) attended the laboratory on five occasions and completed cycling acute exercise for 20 minutes at five intensities (40%, 50%, 60%, 70%, and 80% heart rate reserve (HRR)). At the right carotid artery, center-line velocity and arterial inner diameter waveforms were examined before and immediately after exercise. Based upon the measured data, the classical hemodynamic theory was used to calculate the apparent elasticity and the local hemodynamic variables.

**Results:**

The arterial apparent stiffness and the apparent elastic modulus following acute cycling exercise at 60% to 80% HRR were significantly higher than baseline. The mean center-line velocity accelerated from 50% to 80% HRR, but no intensity of intervention altered mean blood flow. Immediately after intervention, the mean wall shear stress and oscillatory shear index increased.

**Conclusions:**

Aerobic cycling intervention, with intensity from 40% to 80% HRR, did not change the brain blood supply. A bout of cycling intervention decreased apparent elasticity, and there was an intensity-dependent effect on apparent elasticity and hemodynamic variables. This study would provide referable data for the further study on the effects of aerobic exercise on arterial hemodynamics and elasticity and underlying physiological mechanisms.

## 1. Introduction

As a major public health problem, the burden of cardiovascular diseases (CVDs) is increasing. In 2017, the WHO has reported that 17.9 million people died from CVDs each year, representing 31% of all deaths worldwide [1].

Arterial stiffness is an important risk factor for predicting the occurrence and development of cardiovascular events, which reflects the elastic function of the arteries. In addition, hemodynamic variables, including wall shear stress (WSS), oscillatory shear index (OSI), pulsatility index (PI), and blood pressure (BP), induce structural and functional changes in the arteries. As a detection window, common carotid artery collects hemodynamic information from the upstream heart and the downstream cerebrovascular bed, of which the hemodynamic changes play crucial roles in reflecting and regulating cardiovascular health [2].

The article "Acute Effects of Different Intensities of Cycling Acute Exercise on Carotid Arterial Apparent Elasticity and Hemodynamic Variables" was published in 2020. Journal: Biomed Res Int.

Increasing physical activity is one of the population-wide interventions that can be implemented to reduce CVDs. In contrast, excessive exercise may have negative effects and cause vascular diseases [3]. In addition, it is clear that effects of acute endurance and resistance exercise intervention (e.g., cycle exercise and handgrip exercise) on arterial stiffness and hemodynamics contribute to changes in arterial structure and function [4]. Therefore, the effect of exercise on vascular health can be evaluated by observing alterations in arterial stiffness and hemodynamic variables, and it is important to explore the intensity dependence of these variables to provide referable information for making exercise plans.

Previous studies have reported the benefits of regular aerobic exercise on arterial stiffness and blood pressure, whether at moderate or high intensity [5–7]. Conversely, few studies have emerged about the effects of different exercise intensities on stiffness and hemodynamics. The acute effects of different intensities of exercise on arterial stiffness are not consistent in the literature. Boutcher et al. have shown that a bout of acute cycling exercise for 20 min at 60% of maximal oxygen uptake (VO_2max_) did not change arterial stiffness (AIx) in normotensive subjects [8]. However, it was reported that a bout of cycling exercise for 60 min at 65-75% heart rate reserve (HRR) reduced arterial stiffness (PWV) [9], and it was also found that moderate intensity (50%VO_2max_) cycling reduced arterial stiffness compared to low intensity (25%VO_2max_) and high intensity (75%VO_2max_) [10]. On the other hand, most studies on the effects of acute exercise intervention on hemodynamics have focused on common variables, such as blood pressure and shear stress. After acute high-intensity interventions, Babcock et al. have reported that systolic and diastolic pressure increased significantly [11], but another report showed a slight decrease in diastolic blood pressure [12]. After acute exercise at 80% of maximal heart rate (HR_max_), antegrade, retrograde, and mean shear rate increased [13]. During the handgrip exercise, Green et al. found that the antegrade shear stress increased and was positively correlated with the exercise intensity, while the retrograde shear stress did not change significantly [14]. Thus, the hemodynamic results were also controversial.

The article "Acute Effects of Different Intensities of Cycling Acute Exercise on Carotid Arterial Apparent Elasticity and Hemodynamic Variables" was published in 2020. Journal: Biomed Res Int.

In brief, it was impossible to comprehensively compare the results of the previous studies to determine the relationship between arterial hemodynamic response and exercise intensity, due to inadequate exercise intensity and hemodynamic parameters. Therefore, it remains unclear if apparent elasticity and arterial hemodynamic variables (including WSS, OSI, PI, and vascular resistance) change after aerobic exercise intervention at different intensities.

The purpose of this study was to compare the acute effects of different intensities of exercise intervention on carotid arterial stiffness and hemodynamic variables and provide a greater variety of hemodynamic information on the impact of aerobic cycling exercise. Towards this end, it is necessary to set more levels of intensity for intervention and enrich the detection of hemodynamic variables. Exercise interventions were set to five levels, ranging from 40% HRR to 80% HRR, with intervals of 10% HRR in this study. It was hypothesized that there was an intensity-dependent effect on hemodynamic response.

## 2. Methods

### 2.1. Subjects

In this study, 32 healthy young male subjects (age: 19.4 ± 0.6 years; height: 175.1 ± 6.1 cm; weight: 66.72 ± 8.95 kg) were recruited from the community to participate in acute aerobic cycling interventions with five different intensities. The criteria for inclusion were individuals who were not involved in any regular planned exercise program (exercise less than 3 times a week and less than 30 min each time) over the last 6 months. None of the subjects were obese. All subjects had no history of heart disease, hypertension, or other diagnosed cardiovascular or metabolic diseases. Subjects were instructed to avoid smoking, vigorous exercise, and medication or food that affect the cardio- and cerebrovascular function 24 hours before the test.

### 2.2. Ethical Approval

This study adhered to the Declaration of Helsinki (1964) and was approved by the Ethics Committee of Dalian University of Technology. All subjects gave the informed written consent after a detailed description of the study procedures.

### 2.3. Experimental Design

Each subject took part in five trials of different exercise intensities in random order, all of which differed only in intensity. The intensity of exercise was determined by the heart rate reserve (HRR) method. The targeted heart rates were calculated using the Karvonen formula, which is target heart rate = (220 − age − resting heart rate) × exercise intensity (%) + resting heart rate. On the first visit, before baseline measurements, subjects seated quietly for 15 minutes and resting heart rates were measured. The target heart rates for different intensities of exercise were calculated based on the resting heart rates.

The article "Acute Effects of Different Intensities of Cycling Acute Exercise on Carotid Arterial Apparent Elasticity and Hemodynamic Variables" was published in 2020. Journal: Biomed Res Int.

The aerobic cycling intervention protocol is shown in Figure 1. After subjects lay in the supine position for 10 minutes, the arterial inner diameter and center-line blood flow velocity waveforms of the right common carotid artery were measured by color Doppler ultrasound (Prosound Alpha 7, Aloka, Japan). Synchronously, heart rate, brachial systolic pressure (*p*_s_mea_), and diastolic pressure (*p*_d_mea_) were recorded in triplicate, positioned on the left arm, using a cuff-type electronic manometer (Patient Monitor PM8000, Mindray). Then, after a full warm up and brief recovery, the power bike (Powermax VIII, Combi Wellness, Japan) was used by subjects for performing an acute cycling intervention for 20 minutes with a fixed set to 4 kp. During the 20-minute exercise intervention, the cycling speed was monitored and adjusted to keep the heart rate within the required heart rate range. By using an ear-clip heart rate sensor connected to the power bike, heart rate was monitored and transmitted to the power bike's screen in real time. After the cycling intervention, subjects immediately regained the supine position and the assessment of hemodynamics was repeated. In this study, the intensity required in the cycling intervention phase was 40%, 50%, 60%, 70%, and 80% HRR, respectively. To avoid confounding effects, the trials were separated by 7 days.

### 2.4. Calculation of Local Hemodynamics

We followed the methods of Liu et al. to calculate the local apparent arterial stiffness and hemodynamic variables [15].

#### 2.4.1. Blood Pressure (*p*)

In this study, the mean value of the carotid arterial pressure (*p*_m_) and diastolic pressure (*p*_d_) were assumed to be equal to the mean value of the brachial pressure (*p*_m_mea_) and diastolic pressure (*p*_d_mea_), as performed in a previous investigation [16]. The mean arterial pressure (*p*_m_) was calculated using the following equation:

(1) $$\begin{array}{c} p_{\text{m}}=p_{\text{m\_mea}}=p_{\text{d\_mea}}+\frac{1}{3}\left(p_{\text{s\_mea}}-p_{\text{d\_mea}}\right), \end{array}$$

where *p*_s_mea_ is the brachial systolic pressure.

Therefore, the waveforms of *p*_m_ were calibrated using the brachial mean arterial (*p*_m_mea_) and diastolic (*p*_d_mea_) pressure. The maximal value of the carotid arterial pressure waveform was then calculated and assumed to be the carotid arterial systolic pressure (*p*_s_).

The article "Acute Effects of Different Intensities of Cycling Acute Exercise on Carotid Arterial Apparent Elasticity and Hemodynamic Variables" was published in 2020. Journal: Biomed Res Int.

#### 2.4.2. Flow Rate (*Q*)

The flow rate was computed as

(2) $$\begin{array}{c} Q=2\pi {{\overset{\text{\_}}{R}}_{0}}^{2}\int_{0}^{1}y\cdot u\left(y,t\right)dy, \end{array}$$

where *R*_0_ is the average of the radius of the common carotid artery over time during a cardiac cycle. *t* is the period of one cardiac cycle. *y* = *r*/*R*_0_, in which *r* is the radial coordinate. *u*(*y*, *t*) satisfies

(3) $$\begin{array}{c} u\left(y,t\right)=\overset{+\infty }{\underset{n=-\infty }{\sum }}\frac{J_{0}\left(\alpha_{n}j^{3/2}\right)-J_{0}\left(\alpha_{n}j^{3/2}y\right)}{J_{0}\left(\alpha_{n}j^{3/2}\right)-1}u\left(0,\omega_{n}\right)e^{j\omega_{n}t}, \end{array}$$

where *J*_0_ is the 0th-order Bessel function of the first kind and $j=\sqrt{-1}$. *α*_*n*_ is the Womersley number and *n* is the harmonic number. $a_{n}=R_{0}\sqrt{\rho \omega_{n}/\eta }$, in which *ρ* is the density of blood and *η* is blood viscosity. Due to the limited experimental conditions, *η* and *ρ*, in the present study, were taken as the same values for all subjects. *η* = 0.004 Pa · s and *ρ* = 1050 kg/m^3^, respectively. *ω*_*n*_ = 2*nπf* is the angular frequency, and *f* is the base frequency. *u*(0, *ω*_*n*_) is the *n* harmonic component of the measured center-line velocities. The maximal harmonic number *n* was computed as 20 and satisfies

(4) $$\begin{array}{c} u\left(0,t\right)=\overset{+\infty }{\underset{n=-\infty }{\sum }}u\left(0,\omega_{n}\right)e^{j\omega_{n}t}. \end{array}$$

#### 2.4.3. Apparent Elastic Modulus (*E*_p_)

Arterial elastic function reflects the degree of change in arterial volume caused by changes in blood pressure per unit. The apparent elastic modulus was computed as

(5) $$\begin{array}{c} E_{\text{p}}=\frac{p_{\text{s}}-p_{\text{d}}}{R_{\text{s}}-R_{\text{d}}}\cdot R_{\text{d}}. \end{array}$$

#### 2.4.4. Apparent Stiffness Index (*β*)

*β* was calculated as the mean of adjusting arterial compliance for changes in normal stress as follows:

(6) $$\begin{array}{c} \beta =\frac{\ln\left(p_{\text{s}}/p_{\text{d}}\right)}{R_{\text{s}}-R_{\text{d}}}\cdot R_{\text{d}}. \end{array}$$

#### 2.4.5. Wall Shear Stress (WSS)

The blood flowing along the vascular vessel creates a tangential frictional force, known as wall shear stress (*τ*_w_), and was computed as

(7) $$\begin{array}{c} \tau_{\text{w}}=\frac{\eta }{R_{0}}\overset{+\infty }{\underset{n=-\infty }{\sum }}\frac{\alpha_{n}j^{3/2}J_{1}\left(\alpha_{n}j^{3/2}\right)}{J_{0}\left(\alpha_{n}j^{3/2}\right)-1}u\left(0,\omega_{n}\right)e^{j\omega_{n}t}, \end{array}$$

where *J*_1_ is the first-order Bessel function of the first kind.

#### 2.4.6. Oscillatory Shear Index (OSI)

The oscillatory shear index is an index that describes the ratio of the retrograde shear stress to the total shear stress and was defined as

(8) $$\begin{array}{c} \text{OSI}=\frac{1}{2}\left(1-\frac{\left|\int_{0}^{T}\tau_{\text{w}}dt\right|}{\int_{0}^{T}\left|\tau_{\text{w}}\right|dt}\right). \end{array}$$

The article "Acute Effects of Different Intensities of Cycling Acute Exercise on Carotid Arterial Apparent Elasticity and Hemodynamic Variables" was published in 2020. Journal: Biomed Res Int.

#### 2.4.7. Pulsatility Index (PI)

The pulsatility index is used to express the relationship between blood flow pulsation and arterial pulsation and was calculated by the following equation:

(9) $$\begin{array}{c} \text{PI}=\frac{V_{\max}-V_{\min}}{V_{\text{mean}}}, \end{array}$$

where *V*_max_, *V*_min_, and *V*_mean_ are the maximum, minimum, and mean blood center-line velocities, respectively.

#### 2.4.8. Dynamic Resistance (DR)

Dynamic resistance represents the ability of arterial regulation. The dynamic resistance was calculated as follows:

(10) $$\begin{array}{c} \text{DR}=\frac{p_{\text{s}}-p_{\text{d}}}{Q_{\max}-Q_{\min}}, \end{array}$$

where *Q*_max_ and *Q*_min_ are the maximum and minimum value of blood flow rate, respectively.

#### 2.4.9. Peripheral Resistance (*R*_p_)

The peripheral resistance reflects the patency of capillaries in the brain and microcirculation in the intracranial vascular bed and was calculated by the following equation [17]:

(11) $$\begin{array}{c} R_{\text{p}}=\frac{p_{\text{m}}}{Q_{\text{mean}}}, \end{array}$$

where *Q*_mean_ is the mean blood flow rate.

### 2.5. Data Processing and Statistical Analysis

Equations (1)–(11) were programmed by Matlab (The MathWorks R2009b, Inc.), and local hemodynamics was calculated. The waveforms of wall shear stress and velocity in the equation were expanded by Fourier series. All data were presented as the mean ± SD.

GraphPad Prism 8 (GraphPad Software, Inc.) was applied for data statistics and analysis. The one-way ANOVA was performed to assess the differences between baseline and the hemodynamics immediately after exercise with different intensities. When significant differences were detected, LSD was used for post hoc comparisons. The significance level was set at *P* < 0.05.

## 3. Results

### 3.1. Effects of Different Intensities of Acute Cycling on the Elastic Function of Carotid Artery

Figures 2(a) and 2(b) indicate that pressure-strain elastic modulus (*E*_p_) and arterial stiffness index (*β*) at 60%, 70%, and 80% HRR significantly increased after acute cycling exercise compared to those at rest.

The maximal, mean, and minimal diameters at rest and immediately following acute cycling intervention at different intensities are shown in Figures 3(a)–3(c). Compared with at-rest state, the maximal, mean, and minimal diameters were significantly decreased at 50% to 80% HRR immediately after the acute exercise.

The article "Acute Effects of Different Intensities of Cycling Acute Exercise on Carotid Arterial Apparent Elasticity and Hemodynamic Variables" was published in 2020. Journal: Biomed Res Int.

### 3.2. Effects of Different Intensities of Acute Cycling on the Blood Supply to the Brain

Table 1 lists the acute changes in blood supply to the brain at different intensities of acute cycling. Maximum and mean center-line velocities (*V*_max_ and *V*_mean_) increased significantly after exercise intervention compared with rest when the intensity was equal or greater than 50% HRR. Compared with at-rest state, the minimum center-line velocity (*V*_min_) was significantly lower after acute exercise at 60%, 70%, and 80% HRR. The minimum blood flow rate (*Q*_min_) was significantly decreased immediately after acute exercise and showed a negative value when the intensity of cycling was equal or greater than 50% HRR. Compared with at-rest state, the maximum blood flow rate (*Q*_max_) and mean blood flow rate (*Q*_mean_) did not change significantly after any intensity of acute exercise.

### 3.3. Effects of Different Intensities of Acute Cycling on Hemodynamics

As indicated in Figures 4(a)–4(c), immediately after the cycling intervention, the systolic pressure (*p*_s_) was significantly increased at any intensity of exercise. When exercise intensity was 70% HRR or less, the mean blood pressure (*p*_mean_) after acute cycling was higher than that at rest. Compared to the resting state, immediately after acute exercise, the diastolic pressure (*p*_d_) increased significantly when the intensity was not higher than 60% HRR.

As shown in Figures 5(a)–5(c), immediately after any intensities of exercise, the maximal and mean wall shear stress (*τ*_w_max_ and *τ*_w_mean_) were significantly increased than at rest and increased with the increase in intensity. The minimal wall shear stress (*τ*_w_min_) has a negative value and significantly lower than that at rest when the intensity was from 50% to 80% HRR.  Figure 5(d) indicates that the oscillatory shear index (OSI) was significantly higher than the resting value and increased with the increase in intensity of exercise.

Figure 6(a) shows that dynamic resistance (DR) decreased with the increase of exercise intensity and was lower than the resting value immediately after acute cycling intervention. As Figure 6(b) indicated, immediately after acute exercise, peripheral resistance (*R*_p_) decreased significantly when the intensity of exercise was 70% HRR or 80% HRR, compared to that at rest.  Figure 6(c) shows that the greater the intensity of exercise, the greater the pulsatility index (PI). Compared with the resting state, PI increased significantly after acute cycling exercise at 50% to 80% HRR.

## 4. Discussion

In the present study, we evaluated carotid arterial stiffness and hemodynamics responses to different intensities of cycling exercise in healthy young men. Our results confirm previous work, showing that blood flow, wall shear stress (WSS), and systolic blood pressure (*p*_s_) are increased by moderate- and high-intensity aerobic exercise [18, 19]. The novel findings of the current study were as follows. (1) A single bout of cycling exercise resulted in increased carotid artery stiffness (*β*) and elasticity modulus (*E*_p_) with exercise intensity at 60% to 80% HRR and acute constriction of the common carotid artery with exercise intensity higher than 50% HRR. (2) Exercise led to significant increase in the maximal and mean values of center-line velocities (*V*_max_ and *V*_mean_) with exercise intensity at 50% to 80% HRR. However, the maximal and mean values of flow rate (*Q*_max_ and *Q*_mean_) did not respond significantly to the change in intensity. (3) After cycling, the maximal and mean values of wall shear stress (*τ*_w_max_ and *τ*_w_mean_), oscillation shear index (OSI), and pulsatility index (PI) are higher than the resting value and increased with increasing intensity. Dynamic resistance (DR) and peripheral resistance (*R*_p_) decreased with increasing intensity.

The article "Acute Effects of Different Intensities of Cycling Acute Exercise on Carotid Arterial Apparent Elasticity and Hemodynamic Variables" was published in 2020. Journal: Biomed Res Int.

### 4.1. Response of Arterial Elastic Functions to Acute Cycling at Different Intensities

Acute exercise intervention can induce transient changes in arterial function and structure. With different exercise types and intensities, exercise may have different or even opposite effects on the arterial elastic function [20]. Higher arterial stiffness and elastic modulus mean worse arterial elastic function. It was reported that a significant increase in arterial stiffness was observed after high-intensity cycling training [11]. However, studies have found that arterial stiffness decreases or does not change after low- to moderate-intensity aerobic exercise [21, 22]. Sharman et al. recruited 12 male subjects and discussed the systemic and peripheral hemodynamic responses after the cycling exercise intervention. The exercise intensity selected in the study was 50%, 60%, 70%, and 80% of the maximum heart rate, respectively. The study found that the estimated aortic pulse wave velocity increased during exercise, which means an increase in aortic stiffness [23]. In this study, it was found that the elastic function of the common carotid artery decreased significantly at 60%, 70%, and 80% HRR, and the arteries stiffened with the increase of exercise intensity. When the intensity of exercise was 50% to 80% HRR, the diameter of the common carotid artery decreased significantly after acute cycling exercise and decreased with the increase of exercise intensity.

The article "Acute Effects of Different Intensities of Cycling Acute Exercise on Carotid Arterial Apparent Elasticity and Hemodynamic Variables" was published in 2020. Journal: Biomed Res Int.

The buffering capacity of an artery is affected by its structural (wall thickness), functional (stiffness), and geometric characteristics (diameter) [24]. Meanwhile, in order to maintain appropriate blood flow and pressure, arterial elasticity is also regulated by the interaction between vasodilators and vasoconstrictor reflex (controlled by sympathetic nerves) [3]. From a neuroregulatory perspective, during and after exercise, the mechanism for the increased stiffness of common carotid arteries may be tonic contractions of the blood vessels, which can be caused by sympathetic excitation and the related increase in circulating catecholamines [25]. In addition, exercise may also promote the release of endothelin-1, leading to vasoconstriction [26]. In the field of physiology, acute injury to endothelial function, increased markers of oxidative stress, or increased mean arterial blood pressure may be associated with decreased arterial elastic function [12, 27, 28]. Studies suggested that low-intensity exercise may reduce vasoconstriction by inhibiting sympathetic and adrenal hormones [3]. However, high-intensity exercise may lead to increased arterial stiffness and related changes in the structure and function [29]. On the one hand, high-intensity exercise may enhance the activities of the sympathetic nervous system and myogenic response and promote the increase of norepinephrine and blood pressure in plasma; on the other hand, the increase of adverse blood flow induced by high-intensity exercise can promote the production of superoxide and reduce the bioavailability of nitric oxide (NO).

### 4.2. Response of Cerebral Blood Supply to Acute Cycling at Different Intensities

Acute exercise intervention can induce increased human heart rate and accelerated blood flow, which can induce global or local hemodynamic response [4]. At the beginning of exercise, the arterial blood flow and wall shear stress of the moving limbs will increase significantly and continuously increase with the increase of exercise intensity, so as to meet the increased demand of the organs for oxygen [30]. In this study, it was pointed out that there was a positive correlation between *V*_mean_ and exercise intensity. However, no matter how high the exercise intensity was, there was no significant difference in *Q*_mean_ before and after exercise. The brain blood supply functions through 2 pairs of arteries, the internal carotid arteries and vertebral arteries. In healthy people without cardio- or cerebrovascular disease, *Q*_mean_ of the right common carotid artery was considered to be an indicator of blood supply to the brain. Therefore, the results mean that exercise did not alter the blood supply to the brain at 40% to 80% HRR. It was worth noting that with the increase of exercise intensity after exercise, the minimum blood (*Q*_min_) flow was negative, which means that there is a retrograde phenomenon of blood flow after exercise. The occurrence of this phenomenon may be related to the imbalance of endothelium-derived vasoactive factors (i.e., NO and endothelin-1) or may be the result of the combined effects of increased arterial stiffness, decreased diameter, and increased dynamic resistance. The detailed mechanism needs to be studied in longer term experiments.

The article "Acute Effects of Different Intensities of Cycling Acute Exercise on Carotid Arterial Apparent Elasticity and Hemodynamic Variables" was published in 2020. Journal: Biomed Res Int.

### 4.3. Hemodynamic Responses to Acute Cycling at Different Intensities

Systolic blood pressure increased significantly after exercise of all five levels of intensity, but diastolic blood pressure increased immediately after exercise of 40%, 50%, and 60% HRR. There was no significant difference between diastolic blood pressure and resting value when exercise intensity reached 70% and 80% HRR. Previous researches have reported that diastolic blood pressure decreases or does not change, during exercise or in the postexercise period, in normotensive subjects [31]. In this study, acute changes in apparent elasticity and diameter of the arteries may contribute to the increased blood pressure immediately after cycling intervention. In addition, after exercise of 40%-60% HRR, the intensity of exercise may be too low to cause centrally mediated decreases in sympathetic nerve activity. But higher intensity (70%-80% HRR) of exercise may drive activation of local vasodilator mechanisms and reduce signal transduction from sympathetic nerve activation into vasoconstriction. Immediately after exercise, mean blood pressure (*p*_mean_) decreased with the increase of exercise intensity. In this study, *p*_mean_ has been calculated for each heart rate interval with a standard formula. During or after exercise, the rate of the systolic : diastolic changes as the heart rate increases. As a result, *p*_mean_ estimated using the standard formula may be lower than the corrected formula [32]. Considering that systolic blood pressure is not strongly dependent on intensity, it can be speculated that 70% and 80% HRR exercise is better for suppressing negative changes in blood pressure.

*R*_p_ refers to the resistance borne by blood when flowing in the cerebrovascular bed, which is related to blood viscosity and diameter of blood vessels. In the present study, there is no significant difference in subject's baseline physical characteristics. All participants were under 20 years of age and not overweight. They had no history of any disease known to affect the cardio- and cerebrovascular systems. Therefore, the blood viscosity (*η*) was uniformly set as 0.004 Pa·s. It was found that after cycling at 70% and 80% HRR, *R*_p_ was significantly lower than the resting state, indicating that the overall resistance of the intracranial and extracranial peripheral vascular bed could be reduced by higher intensity exercise. DR reflects the relationship between changes in blood pressure and corresponding changes in blood flow. PI reflects the resistance of the vascular bed, and higher PI means lower resistance. This study found that when the intensity of exercise is not less than 40% HRR, DR decreased significantly and is negatively correlated with the intensity. PI increased significantly after acute exercise with 50% HRR or higher intensity. We can assume that when the intensity of exercise is not less than 50% HRR, cycling exercise allows blood flow more easily.

The article "Acute Effects of Different Intensities of Cycling Acute Exercise on Carotid Arterial Apparent Elasticity and Hemodynamic Variables" was published in 2020. Journal: Biomed Res Int.

Wall shear stress (WSS) is defined as the traction force of blood flow on the vascular wall and represents the friction force acting on the vascular endothelium. Studies have shown that WSS plays an important role in the occurrence and development of atherosclerosis, which mainly occurs in areas of low [4]. After exercise training, obvious retrograde blood flow can be observed locally in some arteries, and the magnitude of the retrograde flow is affected by the exercise modes [33]. In this study, the minimum value of WSS (*τ*_w_min_) decreased and was negative, which means that there was retrograde WSS. The occurrence of retrograde WSS implied the phenomenon of retrograde blood flow, which was consistent with *Q*_min_. However, *τ*_w_max_ and *τ*_w_mean_ increased significantly, so it can be considered that the amplitude of increase of WSS in the forward direction is higher than that in the reverse direction, which may be beneficial to the improvement of vascular endothelial function and reduce the risk of atherosclerosis. Whether the oscillatory shear index is a positive or negative regulator of arterial structure and function remains to be determined.

## 5. Conclusions

Our findings demonstrated that arterial stiffness increases immediately after exercise when the intensity is 60% HRR or higher in healthy young men. In contrast, higher intensity was accompanied by lower diastolic blood pressure and vascular bed resistance. There was an intensity-dependent effect on hemodynamic response. However, in this study, no matter how intense the acute cycling exercise was, it did not alter the blood supply to the brain.

## 6. Limitations

There are limitations in this study. First, only the acute effect of exercise with different intensities on carotid arterial elastic function and hemodynamics was investigated and compared (immediately after exercise). There was a lack of follow-up monitoring of the long-term responses of arterial stiffness and hemodynamics after a bout of exercise. Second, we focused only on the effects of acute exercise in healthy people, and future studies could be conducted in people with cardiovascular disease or metabolic syndrome.

The article "Acute Effects of Different Intensities of Cycling Acute Exercise on Carotid Arterial Apparent Elasticity and Hemodynamic Variables" was published in 2020. Journal: Biomed Res Int.

## Figures and Tables

**Figure 1:** Acute aerobic cycling intervention at different intensity protocol.

**Figure 2:** Acute effects of exercise on elastic function at different intensities. (a) Pressure-strain elastic modulus (*E*_p_). (b) Arterial stiffness index (*β*). ^∗^*P* < 0.05 vs. rest.

**Figure 3:** Acute effects of exercise on carotid diameters (*D*) at different intensities. (a) Maximal artery diameters (*D*_max_). (b) Mean artery diameters (*D*_mean_). (c) Minimal artery diameters (*D*_min_). ^∗^*P* < 0.05 vs. rest.

**Figure 4:** Acute effects of exercise on carotid blood pressure (*p*) at different intensities. (a) Systolic blood pressure (*p*_s_). (b) Mean blood pressure (*p*_mean_). (c) Diastolic blood pressure (*p*_d_). ^∗^*P* < 0.05 vs. rest.

**Figure 5:** Acute effects of exercise on carotid wall shear stress (WSS) and oscillatory shear index (OSI) at different intensities. (a) Maximal wall shear stress (*τ*_w_max_). (b) Mean wall shear stress (*τ*_w_mean_). (c) Minimal wall shear stress (*τ*_w_min_). (d) Oscillatory shear index (OSI). ^∗^*P* < 0.05 vs. rest.

**Figure 6:** Acute effects of exercise on (a) carotid dynamic resistance (DR), (b) peripheral resistance (*R*_p_), and (c) pulsatility index (PI) at different intensities. ^∗^*P* < 0.05 vs. rest.

**Table 1:** Effects of different intensities of acute cycling on the blood supply to the brain.

	Rest	Immediately after the cycling intervention at different intensities				
		40%	50%	60%	70%	80%
*V*_max_ (m/s)	0.73 ± 0.12	0.86 ± 0.14	0.91 ± 0.14^∗^	0.91 ± 0.14^∗^	1.03 ± 0.17^∗^	1.06 ± 0.18^∗^
*V*_mean_ (m/s)	0.31 ± 0.03	0.37 ± 0.05	0.39 ± 0.06^∗^	0.39 ± 0.04^∗^	0.43 ± 0.07^∗^	0.44 ± 0.06^∗^
*V*_min_ (m/s)	0.19 ± 0.03	0.18 ± 0.05	0.15 ± 0.09	0.11 ± 0.09^∗^	0.08 ± 0.10^∗^	0.06 ± 0.08^∗^
*Q*_max_ (ml/s)	11.73 ± 2.80	13.27 ± 2.71	12.83 ± 3.43	12.51 ± 3.03	13.59 ± 2.67	13.82 ± 3.10
*Q*_mean_ (ml/s)	3.71 ± 0.63	4.24 ± 0.83	4.10 ± 0.89	3.97 ± 0.77	4.16 ± 0.76	4.15 ± 0.76
*Q*_min_ (ml/s)	0.82 ± 1.22	0.12 ± 1.34^∗^	−0.18 ± 1.66^∗^	−0.75 ± 1.71^∗^	−1.55 ± 1.99^∗^	−2.14 ± 1.99^∗^

Values are means ± SD. *V*_max_: maximal center-line velocity; *V*_mean_: mean center-line velocity; *V*_min_: minimal center-line velocity; *Q*_max_: maximal flow rate; *Q*_mean_: mean flow rate; *Q*_min_: minimal flow rate. ^∗^*P* < 0.05 vs. rest.

The article "Acute Effects of Different Intensities of Cycling Acute Exercise on Carotid Arterial Apparent Elasticity and Hemodynamic Variables" was published in 2020. Journal: Biomed Res Int.

## Data Availability

All data used to support the findings of this study are included within the article.
